The article "Study on Model Iterative Reconstruction Algorithm vs. Filter Back Projection Algorithm for Diagnosis of Acute Cerebral Infarction Using CT Images" was published in 2021. Journal: J Healthc Eng.

# Study on Model Iterative Reconstruction Algorithm vs. Filter Back Projection Algorithm for Diagnosis of Acute Cerebral Infarction Using CT Images

**DOI:** 10.1155/2021/5000102

**Published:** 2021-08-05

**Authors:** Songlin Tang, Yan Liu, Zhifu Wang, Yajie Liu, Huafei Liu

**Affiliations:** ^1^Department of Neurology, The First Affiliated Hospital of Shaoyang College, Shaoyang 422039, Hunan, China; ^2^Department of Imaging, Shaoyang Central Hospital, Shaoyang 422100, Hunan, China

## Abstract

The aim was to explore the application value of computed tomography (CT) perfusion (CTP) imaging based on the iterative model reconstruction (IMR) in the diagnosis of acute cerebral infarction (ACI). 80 patients with ACI, admitted to hospital, were selected as the research objects and divided randomly into a routine treatment group (group A) and a low-dose group (group B) (each group with 40 patients). Patients in group A were scanned at 80 kV–150 mAs, and the traditional filtered back projection (FBP) algorithm was employed to reconstruct the images; besides, 80 kV–30 mAs was adopted to scan the patients in group B, and the images were reconstructed by IMR1, IMR2, IMR3, iDose4 (a kind of hybrid iterative reconstruction technology), and FBP, respectively. The application values of different algorithms were evaluated by CTP based on the collected CTP images of patients and detecting indicators. The results showed that the gray and white matter CT value, SD value, SNR, CNR, and subjective image scores of patients in group B were basically consistent with those of group A (*p* > 0.05) after the IMR1 reconstruction, and the CT and SD of gray and white matter in patients from group B reduced steeply (*p* < 0.05), while SNR and CNR increased dramatically after IMR2 and IMR3 reconstruction in contrast to group A (*p* < 0.05). Furthermore, the cerebral blood volume (CBV), cerebral blood flow (CBF), mean transit time (MTT) of contrast agent, and time to peak (TTP) of contrast agent in patients from group B after iDose4 and IMR reconstruction were basically the same as those of group A (*p* > 0.05). Therefore, IMR combined with low-dose CTP could obtain high-quality CTP images of the brain with stable perfusion indicators and low radiation dose, which could be clinically applied in the diagnosis of ACI.

## 1. Introduction

ACI is a common disease and also known as acute ischemic stroke. Its main feature is that blood clots emerges in the brain blood vessels or various reasons lead to insufficient blood supply to the brain, which causes brain tissue ischemia and hypoxia to result in the irreversible apoptosis which is the main cause of death and disability in the old people [1, 2]. It is of great importance to determine the time window of reperfusion therapy for patients with ACI. Moreover, CTP can determine the core of lesion and ischemic area of patients with ACI to make clinical diagnosis and determine the treatment plan in a relatively short time, so as to avoid the constraints of time window, reduce the mortality and disability rate of patients, and monitor patient's prognosis [3].

The article "Study on Model Iterative Reconstruction Algorithm vs. Filter Back Projection Algorithm for Diagnosis of Acute Cerebral Infarction Using CT Images" was published in 2021. Journal: J Healthc Eng.

Although CTP is irreplaceably featured with the diagnosis of patients with ACI, excessive radiation dose is its biggest shortcoming in the diagnosis. CTP requires continuous and repeated scanning of the target area of the brain, resulting in a huge increase in the X-ray radiation dose received by a patient by comparing with conventional CT. Therefore, reducing radiation dose is an urgent clinical topic in the process of CTP application [4, 5]. The main factors that affect CTP radiation dose are voltage, current, collection time, and frequency. Reducing the scanning time and increasing the scanning interval can reduce the radiation, but its effect is extremely limited. An effective method is to reduce the voltage and current, but it is necessary to pay attention to maintaining the quality stability of the perfusion images. Algorithm reconstruction plays an irreplaceable role in maintaining the quality of perfusion images [6].

FBP has been called the gold standard of CT image reconstruction, and it plays a vital role in CT image reconstruction. The amount of projection data reconstructed by FBP has a positive correlation with the resolution of image space and a negative correlation with the image noise, which affects the radiation dose reduction of CT scanning [7, 8]. In order to ensure the image quality of low-dose radiation CT scanning, scholars have focused on the iterative reconstruction technology of CT images, including the iterative reconstruction in image space (IRIS), adaptive statistical iterative reconstruction technology (AsiR), iDose (a kind of hybrid iterative reconstruction technology), and adaptive iterative dose reduction (AIDR) algorithm [9, 10]. Philips' iDose is taken as an example, which applies a dual-model iterative reconstruction algorithm. First, a data model is reconstructed by FBP, and then, it is identified and denoised through a mathematical model and matrix algebra [11]. However, iDose iterative reconstruction algorithm based on FBP is still a partial iterative algorithm. It still does not considers factors such as system hardware problems and X-ray photonic characteristics, which will affect the image quality, thereby limiting the further reduction of scanning radiation dose. After the iDose, Philips' researchers have further developed IMR (a fully iterative reconstruction technology that does not contain FBP components). The mechanism of IMR is to continuously optimize an image and data statistical model and a system model in the image and data space, so as to achieve the objective of denoising. Compared with iDose, IMR can not only reduce noise but also improve the resolution of the image [6, 12, 13].

The article "Study on Model Iterative Reconstruction Algorithm vs. Filter Back Projection Algorithm for Diagnosis of Acute Cerebral Infarction Using CT Images" was published in 2021. Journal: J Healthc Eng.

In summary, the combination of IMR and low-dose CT can achieve the optimization of CTP radiation dose and image quality. This study would explore the application value of IMR-based CTP in the diagnosis of ACI, aiming to provide reliable basic data for clinical applications.

## 2. Materials and Methods

### 2.1. Establishment of Research Objects

80 patients with ACI, who were admitted in hospital, were selected as the research objects. The criteria for inclusion were defined to include patients suffered from ACI, were 18–80 years old, and had signed the informed consents. The criteria for exclusion were defined to contain patients suffered from severe cardiovascular and cerebrovascular diseases, were allergic to the iodine contrast agent, were pregnant or in the lactation period, and had received the arterial stent implantation in the brain. This study had been approved by the ethics committee of hospital. The research objects in the experiment were grouped randomly into group A and B. The tube current in patients of group A was 150 mAs detected by CT, and the tube current of patients in group B was 30 mAs. The FBP image reconstruction was adopted for patients in group A, and FBP, iDose4, IMR1, IMR2, and IMR3 were employed to reconstruct the images of the patients in group B.

### 2.2. Computed Tomography Scanning and Methods

Brilliance iCT Elite CT machine was used for CT scanning. The tube current of patients in group A was 150 mAs, tube current of patients in group B was 30 mAs, tube voltage of patients in both groups was 80 kV, rotation time was 0.33 s, and both of layer thickness and spacing were 5 mm. A double-tube high pressure syringe was applied to inject the contrast agent. After the contrast agent was injected for 4 seconds, it was time to scan. The scan time was 2 seconds, and scanning was repeated 25 times, so the total scan time was 50 seconds. The image reconstruction indicators of FBP and iDose were all standard, and those of IMR1, IMR2, and IMR3 were all normal.

### 2.3. Image Postprocessing

The original image of CTP was transmitted to the workstation (Extend Brilliance Workspace, Philips Healthcare), and the Brain Perfusion software was employed to form a pseudocolor perfusion image of CBF, CBV, MTT, and TTP.

### 2.4. Analysis on the Quality of Images and Objective Evaluation

First, the CT value of white and gray matter on the instantaneous maximum density projection image was measured, and SD of the CT value was regarded as the image noise to calculate the SNR and CNR. The calculation equations were shown as follows. SNR = CT/SD and CNR = (gray matter CT value − white matter of CT value)/(white matter of SD^2^ + gray matter of SD^2^). Second, the values of CBF, CBV, MTT, and TTP were recorded on each pseudocolor image.

The article "Study on Model Iterative Reconstruction Algorithm vs. Filter Back Projection Algorithm for Diagnosis of Acute Cerebral Infarction Using CT Images" was published in 2021. Journal: J Healthc Eng.

### 2.5. Subjective Evaluation of Image Quality Analysis

The 3-level scoring method was for the subjective evaluation standard, with 2 points for good quality, 1 point for average quality, and 0 points for bad quality. The subjective evaluation criteria included the difference of gray and white matter perfusion value on the perfusion pseudocolor image, difference between the focal ischemia and normal tissue, homogeneity of image, contrast of infarction, contour, degrees of concentration and dispersion, and presence or absence of artifacts. The highest score was 8; a score greater than 6 indicated an image with high quality, a score of 3–6 meant a medium-quality image, and a score less than 3 indicated an image of poor quality.

### 2.6. Statistical Analysis

SPSS22.0 was used for statistical analysis of the data. The subjective scores of images from patients in each group were compared by the rank sum test, the variance was employed to analyze the perfusion indicators, CT value, SD value, SNR, and CNR of gray and white matter, and the independent sample *t*-test was applied to the pairwise comparison between groups. *P* < 0.05 meant that there was statistically significant difference.

## 3. Results

### 3.1. Objective Indicators

As given in Table 1, there were the statistically substantial overall differences in the CT value, SD value, SNR, and CNR of gray and white matter among patients from the two groups through the 6 reconstruction methods (*p* < 0.05) after the variance analysis.  Figure 1 shows the CT images processed by different reconstruction methods, including the images of group A reconstructed by FBP, and the images of group B reconstructed by FBP, iDose4, IMR1, IMR2, and IMR3, respectively. It was found that the images with high current were relatively clear (A-FBP), while the CT images obtained by different reconstruction algorithms in group B were slightly different in quality. The reconstructed images of FBP, IMR1, IMR2, and IMR3 were relatively clear, but the reconstructed images of iDose4 were quite fuzzy, which was not good for observation.

### 3.2. Computed Tomography Values of Gray and White Matter in the Brain

Table 1 and Figure 2 show that the CT values of gray and white matter reconstructed by FBP in patients from group A were 56.23 ± 2.45 Hu and 36.23 ± 2.12 Hu, respectively. In contrast to group A, the obtained CT values of gray and white matter reconstructed by FBP and iDose4 increased dramatically in patients of group B (*p* < 0.05); there were no obvious differences in CT values of gray and white matter reconstructed by IMR1 in patients from group B (*p* > 0.05); the CT value of gray matter reconstructed by IMR2 reduced sharply (*p* < 0.05), but the value of CT in white matter was not considerably different (*p* > 0.05); and the values of CT in gray and white matter reconstructed by IMR3 reduced hugely both (*p* < 0.05).

The article "Study on Model Iterative Reconstruction Algorithm vs. Filter Back Projection Algorithm for Diagnosis of Acute Cerebral Infarction Using CT Images" was published in 2021. Journal: J Healthc Eng.

### 3.3. Standard Deviation Values of Gray and White Matter in the Brain

Table 1 and Figure 3 reveal that the values of SD in gray and white matter reconstructed by FBP were 7.82 ± 1.43 Hu and 5.21 ± 0.98 Hu in patients from group A, respectively. By comparing with group A, the SD values of gray and white matter obtained from FBP and iDose4 image reconstruction increased markedly in patients from group B (*p* < 0.05); the values of SD in gray and white matter reconstructed by IMR1 were not significantly different (*p* > 0.05); and the SD values of gray and white matter reconstructed by IMR2 and IMR3 reduced extremely (*p* < 0.05).

### 3.4. The Values of Signal-to-Noise Ratio in Gray and White Matter from the Brain

Table 1 and Figure 4 indicate that the values of SNR in gray and white matter reconstructed by FBP in patients from group A were 9.41 ± 1.53 and 10.06 ± 1.32, respectively. Besides, the SNR values of gray and white matter reconstructed by FBP and iDose4 decreased enormously in patients from group B compared with those of group A (*p* < 0.05); the SNR of gray matter did not change significantly under the reconstruction of IMR1 (*p* > 0.05), but the white matter SNR value rose dramatically (*p* < 0.05); and the SNR values of gray and white matter reconstructed by IMR2 and IMR3 grew hugely in patients from group B.

### 3.5. The Values of Contrast-to-Noise Ratio in Gray and White Matter from the Brain

Table 1 and Figure 5 show that the CNR of gray matter in patients from group A was 0.40 ± 0.09 after the reconstruction. The CNR of gray matter reconstructed by FBP and iDose4 dropped extremely in patients from group B (*p* < 0.05) compared with that of group A; there was no great difference in the CNR of patients from group B after IMR1 reconstruction (*p* > 0.05); besides, CNR of gray matter increased dramatically in patients from group B after the reconstruction of IMR2 and IMR3 (*p* < 0.05).

### 3.6. Comparison of Subjective Indicators

The subjective score of FBP and iDose4 image reconstruction was 0 in patients of group B, which could not meet the standard of clinical diagnosis. The subjective scores of FBP reconstruction in patients of group A and IMRE1, IMR2, and IMR3 reconstruction in patients of group B were 7.45 ± 0.34, 7.84 ± 0.84, 7.29 ± 0.62, and 7.34 ± 0.67, respectively. There were no huge differences in the subjective scores of image quality among patients from the two groups after multiple rank sum tests (*χ*^2^ = 0.78 and *p* = 0.92).

The article "Study on Model Iterative Reconstruction Algorithm vs. Filter Back Projection Algorithm for Diagnosis of Acute Cerebral Infarction Using CT Images" was published in 2021. Journal: J Healthc Eng.

### 3.7. Comparison on the Values of Perfusion Indicators

Table 2 presents that there were statistically obvious differences in CBV of white matter and CBF and MTT of gray matter among patients in the two groups under the six reconstruction methods (*p* < 0.05) based on the analysis of variance. In addition, the overall differences of white matter CBV and gray matter TPP were statistically marked among patients in the two groups under the six reconstruction methods (*p* < 0.05).

### 3.8. The Values of Cerebral Blood Volume in the Gray and White Matter

As given in Table 2 and Figure 6, CBV of gray and white matter reconstructed by FBP was 5.08 ± 0.42 mL/100 g and 3.12 ± 0.23 mL/100 g in patients of group A, respectively. In contrast to group A, CBV of gray and white matter reconstructed by iDose4, IMR1, IMR2, and IMR3 had no obvious difference (*p* > 0.05) and CBV of white matter showed no obvious difference in patients from group B (*P* > 0.05), while those reconstructed by FBP reduced steeply (*p* < 0.05).

### 3.9. The Values of Cerebral Blood Flow in the Gray and White Matter

As given in Table 2 and Figure 7, the CBF of gray and white matter reconstructed by FBP in patients from group A was 54.23 ± 4.97 mL/100 g/min and 23.32 ± 2.16 mL/100 g/min, respectively. In contrast to group A, there was no considerable difference in CBF of gray and white matter in patients from group B under the reconstruction of iDose4, IMR1, IMR2, and IMR3 (*P* > 0.05), while the CBF of gray and white matter reconstructed by FBP increased substantially (*p* < 0.05).

### 3.10. The Values of Mean Transit Time in the Gray and White Matter

As given in Table 2 and Figure 8, the values of MTT in gray and white matter reconstructed by FBP in patients from group A were 5.65 ± 0.76 seconds and 7.38 ± 1.12 seconds, respectively. In contrast to group A, the MTT values of gray and white matter reconstructed by FBP and iDose4 rose remarkably in patients from group B (*p* < 0.05), while there were no marked differences in the values of MTT reconstructed by IMR1, IMR2, and IMR3 (*p* > 0.05).

### 3.11. Computed Tomography Perfusion Image Example

Figure 9 shows the CT images of ACI. To be specific, Figure 9(a) is the CT image and Figure 9(b) is the CTP image. It was found that CTP could present richer intracranial information by comparing with CT, which was beneficial to diagnose accurately the patient's lesions.

The article "Study on Model Iterative Reconstruction Algorithm vs. Filter Back Projection Algorithm for Diagnosis of Acute Cerebral Infarction Using CT Images" was published in 2021. Journal: J Healthc Eng.

## 4. Discussion

The normal physiological activity of brain tissues depends on certain blood oxygen supply, and the compensatory contraction of capillary smooth muscle and small artery can alleviate the limited fluctuation of cerebral blood perfusion pressure, so as to maintain basically stable cerebral blood flow [14]. When the reduction in perfusion pressure is less than the circulating reserve capacity of the brain, CBF expresses to be normal or a slight decrease, and CBV often increases at this moment due to arteriolar and capillary dilatation. When the decrease of CBF is greater than that of cerebral circulation reserve force, neurons absorb excess glucose and increase oxygen content to maintain normal cell physiological metabolism. At this time, CBF falls below the threshold of electrical failure, so CBF reduces significantly and CBV is normal or decreases. With the continuous decline of CBF, the metabolism level in the brain changes dramatically, the balance of various substances is disrupted, and there is irreversible apoptosis in neurons, namely, ACI [15], with CBF and CBV both dropping obviously.

CTP requires continuous repeated scanning of the target area, so the radiation dose of a patient is higher enormously than that of CT scanning. Therefore, how to reduce the radiation dose of CTP has been attracting the attention of scholars. The traditional methods for radiation reduction include reducing tube voltage, tube current, and acquisition time and frequency, but these measures are easy to increase image noise. With the application of IMR, the image quality can be guaranteed within the maximum range, thus making the traditional methods well applied [16]. In this study, patients with the CTP scanning mode of 80 kV–150 mAs routine dose combined with FBP image reconstruction were regarded as group A to evaluate the changing patterns of each indicator of gray and white matter in patients from group B under different image reconstruction methods. The results indicated that FBP was for reconstruction in the mode of low dose, and the average CT values of gray and white matter in patients from group B were 40% and 55% higher than that of group A, respectively. Moreover, the average CT values of gray and white matter in patients from group B increased by 20% and 28% after the iDose4 reconstruction, respectively. Therefore, the above data could determine that FBP and iDose4 reconstruction were not suitable for the image reconstruction of the low-dose scanning mode. On the contrary, there was no obvious change in the CT value of gray and white matter in the brain with the application of IMR, the CT value of gray and white matter reconstructed by IMR1 in patients of group B had no great difference from those of group A, the CT value reconstructed by IMR2 in patients of group B was at the middle level, and the CT value reconstructed by IMR3 in patients of group B was less than that of group A. This was related to the superior noise reduction function of IMR, making the CT value of gray and white matter return to normal or even lower than the normal value. Previous studies have shown that IMR has an excellent image noise reduction capability and can also improve image resolution [17]. In addition, studies have indicated that the average image noise and CNR under IMR reconstruction are superior markedly to hybrid iterative reconstruction and FBP technology, and IMR improves remarkably the image quality under low-tube voltage that especially helps to promote the display effect of distal vessels [18]. This is consistent with the results of this study.

The article "Study on Model Iterative Reconstruction Algorithm vs. Filter Back Projection Algorithm for Diagnosis of Acute Cerebral Infarction Using CT Images" was published in 2021. Journal: J Healthc Eng.

## 5. Conclusion

The advantages of the IMR full-model iterative reconstruction algorithm in CTP image reconstruction were verified by comparing with low and conventional dose CTP. The results showed that IMR could ensure the quality of CT images under lower dose of radiation and complete the diagnosis of patients with ACI compared with FBP and iDose4, which could be promoted clinically. Therefore, a new direction was provided by this study for the diagnosis of patients with ACI, and the safety of patients was greatly enhanced during examination. The shortcoming of this study was that it had not been compared with other imaging methods, leading to a relatively single standard for judgment.

## Figures and Tables

**Figure 1:** The processing results of CT image under different reconstruction methods. (a) A-FBP. (b) B-FBP. (c) B-iDose4. (d) B-IMR1. (e) B-IMR2. (f) B-IMR3.

**Figure 2:** Statistical results of CT values of gray and white matter in the brain among patients from groups A and B by different reconstruction methods. A and B are the statistical results of gray and white matter in patients from both groups under various reconstruction methods, respectively. ^*∗*^CT value of patients from group B was dramatically different compared with group A (*p* < 0.05).

**Figure 3:** Statistical results of SD values of gray and white matter in the brain among patients from groups A and B by different reconstruction methods. A and B are the statistical results of gray and white matter in patients from the two groups under various reconstruction methods, respectively. ^*∗*^The SD value of patients from group B was different greatly in contrast to group A (*p* < 0.05).

The article "Study on Model Iterative Reconstruction Algorithm vs. Filter Back Projection Algorithm for Diagnosis of Acute Cerebral Infarction Using CT Images" was published in 2021. Journal: J Healthc Eng.

**Figure 4:** Statistical results of SNR values of gray and white matter in the brain among patients from groups A and B by different reconstruction methods. A is the statistical result of gray matter in patients from the two groups under various reconstruction methods; B is the statistical result of white matter in patients from the two groups under different reconstruction methods. ^*∗*^The SNR value of patients from group B was different obviously compared to group A (*p* < 0.05).

**Figure 5:** Statistical results of CNR of gray matter in the brain among patients from both groups by various reconstruction methods. ^*∗*^The CNR value of group B was different hugely from that of group A (*p* < 0.05).

**Figure 6:** Statistical results of CBV of gray and white matter in the brain among patients from groups A and B under the six reconstruction methods. A is the statistical result of gray matter in patients from the two groups under various reconstruction methods; B is the statistical result of white matter in patients from the two groups under different reconstruction methods. ^*∗*^The CBV value of patients from group B was different considerably by comparing with group A (*p* < 0.05).

**Figure 7:** Statistical results of CBF of gray and white matter among patients from the two groups under different reconstruction methods. A is the statistical result of gray matter in patients from the two groups under the six reconstruction methods; B is the statistical result of white matter in patients from the two groups under different reconstruction methods. ^*∗*^The CBF value of patients from group B had a significant difference compared with group A (*p* < 0.05).

**Figure 8:** Statistical results of MTT of gray and white matter among patients from both groups under the six reconstruction methods. A and B are the statistical results of gray and white matter in patients from the two groups under the six reconstruction methods, respectively. ^*∗*^The MTT value of patients from group B had an obvious difference compared with group A (*p* < 0.05).

**Figure 9:** The (a) CT and (b) CTP images of ACI.

**Table 1:** Comparison results of objective values of image quality among patients from the two groups.

Group	Reconstruction methods		CT (Hu)	SD (Hu)	SNR	CNR
Group A	FBP	Gray matter	56.23 ± 2.45	7.82 ± 1.43	9.41 ± 1.53	0.40 ± 0.09
		White matter	36.23 ± 2.12	5.21 ± 0.98	10.06 ± 1.32	

Group B	FBP	Gray matter	78.69 ± 3.12	12.43 ± 1.54	7.83 ± 0.93	0.21 ± 0.03
		White matter	57.12 ± 2.56	9.26 ± 0.98	7.82 ± 0.72	
	iDose4	Gray matter	65.98 ± 3.12	10.79 ± 1.87	8.21 ± 1.10	0.24 ± 0.02
		White matter	48.34 ± 2.17	8.15 ± 0.85	7.73 ± 0.91	
	IMR1	Gray matter	55.43 ± 3.45	7.24 ± 1.27	10.52 ± 2.13	0.42 ± 0.06
		White matter	38.63 ± 1.91	4.83 ± 0.62	10.98 ± 1.17	
	IMR2	Gray matter	53.24 ± 3.19	6.39 ± 1.28	11.23 ± 2.15	0.57 ± 0.11
		White matter	37.03 ± 4.23	4.97 ± 0.92	11.83 ± 1.86	
	IMR3	Gray matter	52.34 ± 3.92	6.82 ± 1.97	11.65 ± 2.31	0.68 ± 0.21
		White matter	34.61 ± 1.97	3.94 ± 0.82	12.82 ± 1.91	

* Z*		Gray matter	234.96	70.98	36.87	65.14
		White matter	267.25	235.87	75.61	

*p*		Gray matter	<0.001	<0.001	<0.001	<0.001
		White matter	<0.001	<0.001	<0.001	

The article "Study on Model Iterative Reconstruction Algorithm vs. Filter Back Projection Algorithm for Diagnosis of Acute Cerebral Infarction Using CT Images" was published in 2021. Journal: J Healthc Eng.

**Table 2:** Comparison results of perfusion indicators in gray and white matter among patients in the two groups.

Group	Reconstruction methods		CBV (mL/100 g)	CBF (mL/100 g/min)	MTT (s)	TTP (s)
A	FBP	Gray matter	5.08 ± 0.42	54.23 ± 4.97	5.65 ± 0.76	18.65 ± 2.87
		White matter	3.12 ± 0.23	23.32 ± 2.16	7.38 ± 1.12	19.86 ± 2.97

B	FBP	Gray matter	4.76 ± 0.45	61.65 ± 8.32	8.23 ± 1.98	18.74 ± 2.31
		White matter	3.16 ± 0.72	31.54 ± 3.21	11.76 ± 2.12	19.23 ± 2.76
	iDose4	Gray matter	4.98 ± 0.47	53.09 ± 3.97	6.54 ± 1.19	18.54 ± 2.13
		White matter	3.17 ± 0.64	25.76 ± 2.96	10.09 ± 2.01	19.76 ± 3.21
	IMR1	Gray matter	5.32 ± 0.71	51.85 ± 3.21	6.21 ± 0.87	18.65 ± 2.45
		White matter	3.16 ± 0.42	23.76 ± 2.93	7.86 ± 1.32	19.93 ± 2.87
	IMR2	Gray matter	5.54 ± 0.89	51.23 ± 3.63	6.26 ± 0.76	18.65 ± 2.52
		White matter	3.21 ± 0.41	23.67 ± 2.87	7.63 ± 1.06	19.78 ± 2.76
	IMR3	Gray matter	5.39 ± 0.75	52.98 ± 5.87	6.24 ± 0.52	18.76 ± 2.61
		White matter	3.23 ± 0.51	22.54 ± 2.12	7.80 ± 1.13	19.72 ± 2.84

*Z*		Gray matter	5.42	4.87	18.65	0.008
		White matter	0.8	12.43	39.76	0.5

*p*		Gray matter	<0.001	0.001	<0.001	1.8
		White matter	0.72	<0.001	<0.001	0.93

## Data Availability

The data used to support the findings of this study are available from the corresponding author upon request.
